The article "Analysis of Extended Resection of Limb Soft Tissue Leiomyosarcoma" was retracted in 2024. Reasons: suspected computer-generated content; unreliable results or conclusions; concerns about the data; concerns about the results or conclusions.

# Analysis of Extended Resection of Limb Soft Tissue Leiomyosarcoma

**DOI:** 10.1155/2021/2106972

**Published:** 2021-08-03

**Authors:** Qiang Liu, Lijun Tang, Xinhua Hu, Jianxing Ye, Pengcheng Liang, Adriana C. Panayi, Shuhua Wang, Jingde Deng

**Affiliations:** ^1^Department of Orthopedics, Jiangxi Province Xing Guo People's Hospital, Wenming 699th Road, Xingguo, 342400 Jiangxi Province, China; ^2^Department of Rehabilitation Medicine, Jiangxi Province Xingg Guo People's Hospital, Wenming 699th Road, Xingguo, 342400 Jiangxi Province, China; ^3^Division of Plastic Surgery, Division of Plastic Surgery, Brigham and Women's Hospital, Harvard Medical School, Boston, Massachusetts, USA

## Abstract

Leiomyosarcoma is an uncommon soft tissue sarcoma that composed of malignant mesenchymal cells with distinct features of the smooth muscle lineage. Typically affects the uterus and gastrointestinal tract, it can rarely be seen in large blood vessels, lymphatic and glandular duts, the mesentery, the omentum, retroperitoneum, and limbs. Occurrence is particularly rare in the limb region. Retrospective study based on patient records and postoperative pathological histological features. Four patients with limb leiomyosarcoma that were operated between 2016 and 2020 were included, three of them arising in the subcutis of the thigh region and one in cubitus. Extend resection with satisfactory outcomes is reported. Pathological examination showed that masses were composed of a fascicular arrangement of hyperchromatic spindle-shaped cells, characterized by the proliferation of epithelioid cells with eosinophilic cytoplasm for epithelioid leiomyosarcoma. Leiomyosarcomas that arise in the soft tissue, although rare, should be differentiated from other lesions, such as neurilemoma, neurofibroma, liomyoma,lipomyoma, synoviosarcoma, rhabdomyosarcoma, malignant fibrous histiotoma, and malignant neurinoma.

## 1. Introduction

Leiomyosarcoma is an uncommon soft tissue sarcoma composed of malignant mesenchymal cells showing distinct features of a smooth muscle lineage. It usually affects the uterus and gastrointestinal tract but that may be also found in less common sites including large blood vessels, lymphatic and glandular duts, the mesentery, onmentum, and retroperitoneum as well as the limbs. However, the limb region is a rare location [1]. Leiomyosarcomas of the cubitus and subcutis of the thigh region are very infrequent occurrences. Preoperative diagnosis of leiomyosarcoma is challenging because of nonspecific symptoms and a rapidly enlarging mass, and therefore, it mainly depends on postoperative pathological examination. The histological grade, tumor size, and tumor depth are the three major clinical pathologic factors for the prognosis of leiomyosarcoma. Around 90% of leiomyosarcomas are reported to be moderate to high grade [2]. Herein, we report four cases of leiomyosarcoma and discuss possible differential diagnoses.

## 2. Materials and Methods

Four patients with limb leiomyosarcomas based on patient records and postoperative pathological histological features were included in this retrospective study between June 2016 and June 2020.There were 3 males and 1 female with an average age of 41.5 years (21–70 years). All the cases whose primary symptom was asymptomatic except slowly enlarging painless soft tissue masses. The course of the disease was 0.5 year to 2years.Three of them arising in the subcutis of the thigh region, one in cubitus. The masses range from 2 to 8 cm in diameter. Gross total extended resections with 3-5 cm of normal tissue around the tumor and wide negative margins by intraoperative frozen sections were given for all patients. All the patients were primary tumors. And one patient with pulmonary metastasis later was managed with chemotherapy. Follow-up times are from 12 to 36 months (Table 1). All patients provided informed consent preoperatively.

## 3. Result

The postoperative course was uneventful, and functional exercises were progressively started with the help of rehabilitation therapist. Three of the patients had an uncomplicated recovery and showed no evidence of recurrence or metastases. The patient with pulmonary metastasis survived with 2 years of postoperation (Table 1). Typical case is illustrated in pictures at the end of the article (Figures 1(a)–1(e).

## 4. Discussion

Most leiomyosarcomas (LMS) are located in the mesentery, omentum majus, and retroperitoneum, with rare reports in the somatic soft tissue. LMS account for about 10%-15% of limb sarcomas, with predilection for the lower limbs, especially the proximal limb. This may be related to the abundant vasalium in the proximal limb [3]. The incidence of deep bone invasion by LMS in the somatic soft tissue is estimated to be approximately 10%, as first described by Evans in 1965 [4]. Fortunately, there were no deep bone invasions by LMS for the four patients. LMS in the somatic soft tissue most commonly occur in middle-aged and elderly patients with no obvious sex ratio correlations.

Causal factors have been identified for the etiology. A high rate of LMS in somatic soft tissues has been reported in acquired immunodeficiency syndrome (AIDS) and after kidney or liver transplantation. Smooth muscle cells infected by Epstein-Barr virus may be associated with tumor pathogenesis [5]. Hematogenous spread is a frequent event in the LMS of soft tissue, with the lung the most common site of metastasis. Clinical presentation is asymptomatic except slowly enlarging painless soft tissue masses. Enlarged lymph nodes in advanced cancer have been reported [6]. Both reported cases suffered a rapidly progressive lesion which was asymptomatic that vary from 0.5 year to 2 years. Surgical resection is the essential treatment of patients with LMS localized in the somatic soft tissue. The standard surgical procedure involves a complete excision with 3-5 cm of the normal tissue around the tumor and wide negative margins by intraoperative frozen sections, which is the most important prognostic factor for survival, with or without adjuvant chemotherapy and radiation therapy. One patient with pulmonary metastasis preoperation was managed with chemotherapy in our research. LMS localized in the somatic soft tissue have better overall survival than those arising in the retroperitoneum [7].

Iconography examination plays an important role in diagnosing LMS of the soft tissue. MRI images show irregular masses with poor defined boundaries and no obvious capsule surrounding the lesion. Small areas of necrotic cystic degeneration can also be seen within the tumor. Most lesions show nonuniform equisignal on T1WI and patchy high signal on T2WI. Lesions show significantly inhomogeneous enhancement, with a patchy area of low signal and no obvious enhancement in the center of the lesion [8]. CT imaging helped us identify whether there was any bone destruction adjacent to the tumor.

Although imaging examination help for LMS identification in the soft tissue, definite diagnosis depends on postoperative pathological histological features. ELMS of the soft tissue composed of cells showing distinct features of the smooth muscle lineage, which have been characterized as intersecting, sharply marginated fascicles of spindle cells with abundant eosinophilic cytoplasm, and elongated and hyperchromatic nuclei [9]. Proliferation of epithelioid cells with eosinophilic cytoplasm is seen in epithelioid leiomyosarcoma [10]. Immunohistochemical staining showed that vimentin, desmin, SMA, Ki-67, and HHF-35 are positive.

LMS of the soft tissue should be differentiated from benign tumors such as neurilemomas and neurofibromas. If a benign tumor is misdiagnosed preoperatively, local recurrence can occur due to incomplete resection. This can be found to grow along the peripheral nerve and the well-defined margins of benign neurogenic tumors and moderately to significantly enhanced and capsular for the parenchyma of the LMS of the soft tissue, which may help to differentiated from benign tumors [11].

Secondly, there is need to exclude important likely differential diagnosis of LMS in the soft tissue such as synoviosarcoma, rhabdomyosarcoma, malignant fibrous histiotoma, and malignant neurinoma. Synoviosarcoma mainly occurs in young adults (20 to 40 year olds). Localization of synoviosarcoma is mostly around the joints and is closely related to the joint capsule, peritendineum, and adjacent bone. The incidence of bone destruction is greater than 20%, which is higher than LMS in the soft tissue [12]. Rhabdomyosarcoma located in the muscle is another soft tissue malignant tumor that may be misdiagnosed as LMS. It is composed of cells with distinct features of variously differentiated rhabdomyoblasts. Enhancement scans show an unenhanced necrotic area alternated with the enhanced tumor parenchymal region. Necrosis, hemorrhage, calcification, and bone destruction of this tumor is very rare [13]. Other soft tissue malignant tumors that should be distinguished from LMS are malignant fibrous histiotomas, in which various cells can be seen, including mononuclear and multinuclear giant cells and xanthoma cells. Malignant fibrous histiotoma cells arrange radially with inflammatory cells, such as lymphocytes, plasmocytes, and eosinophils. Malignant neurinoma is another malignant mass that can be potentially confused with LMS. The cells of malignant neurinoma are disordered and pleomorphic [14]. The typical histologic pattern of malignant neurinoma is that of plexiform neurofibroma and necrotic lesions surrounded by palisading tumor cells.

Besides, LMS should be differentiated from some other tumors of the limb region. Among the tumors of the limb region that can be confused with LMS are liomyoma and lipomyoma. We can find the difference between the LMS and liomyoma from the invasion, cell atypia, nuclear division, and focal necrosis. Lipomyoma is a common lobulated soft tissue benign tumor composed of mature adipocyte showing distinct features of the mesenchymal tissue.

In conclusion, we describe four cases of LMS arising from the limb region. There are no clear diagnostic criteria for LMS, and diagnosis should be made from the microscopical and histopathological features as well as imaging examinations. LMS should be considered in the differential diagnosis of some lesions including neurilemoma, neurofibroma, liomyoma, lipomyoma, synoviosarcoma, rhabdomyosarcoma, malignant fibrous histiotoma, and malignant neurinoma. We emphasize the potential for malignant transformation of ELMS, highlighting the need for prompt extended resection and close follow-up in their management.

## Figures and Tables

**Figure 1:** A 70-year-old man presented with a three-month history of a soft tissue mass in the subcutis of the left thigh. (a). Magnetic resonance imaging (MRI) revealed a fusiform mass shadow on the subcutis of the left thigh and diffusion-weighted imaging showing high signal. (b). Magnetic resonance imaging (MRI) revealed T1WI sequencing showing low signal. (c). Magnetic resonance imaging (MRI) revealed enhancement scan that showed lesion which was significantly intensify. (d). Histologic features of the lesion showed that the tumor was composed of densely arranged, abundant spindle cells with nuclei that were mild to moderately atypical, and proliferation of epithelioid cells(HE, ×200). (e). Tumor cells showing diffuse immunohistochemical positivity for SMA.

**Table 1:** Demographics of the patients and follow-up data.

Case	Gender (M/F)	Age (year)	Site	Course (year)	Max diameter (cm)	Therapies	Follow-up
1	M	70	Left thigh	0.5	7	Extended resection+chemotherapy	Survive with 2 years
2	M	35	Right cubitus	1	3	Extended resection	No recurrence or metastases 2 years
3	M	21	Right thigh	1.2	8	Extended resection	No recurrence or metastases 1.5 years
4	F	40	Right thigh	2	6	Extended resection	No recurrence or metastases 3 years

## Data Availability

The data analyzed during the current study are available from the corresponding author on reasonable request.
